# Acaricide Residues in Laying Hens Naturally Infested by Red Mite *Dermanyssus gallinae*

**DOI:** 10.1371/journal.pone.0031795

**Published:** 2012-02-21

**Authors:** Marianna Marangi, Vincenzo Morelli, Sandra Pati, Antonio Camarda, Maria Assunta Cafiero, Annunziata Giangaspero

**Affiliations:** 1 Dipartimento di Scienze delle Produzioni, dell'Ingegneria e della Meccanica e dell'Economia Applicate ai Sistemi Agro-Zootecnici, University of Foggia, Foggia, Italy; 2 Laboratori Bonassisa, Consorzio ASI, Foggia, Italy; 3 Dipartimento di Scienze degli Alimenti, University of Foggia, Foggia, Italy; 4 Dipartimento di Sanità Pubblica e Zootecnia, University of Bari, Bari, Italy; 5 Istituto Zooprofilattico Sperimentale della Puglia e Basilicata, Foggia, Italy; Auburn University, United States of America

## Abstract

In the poultry industry, control of the red mite *D. gallinae* primarily relies worldwide on acaricides registered for use in agriculture or for livestock, and those most widely used are carbamates, followed by amidines, pyrethroids and organophosphates. Due to the repeated use of acaricides - sometimes in high concentrations - to control infestation, red mites may become resistant, and acaricides may accumulate in chicken organs and tissues, and also in eggs. To highlight some situations of misuse/abuse of chemicals and of risk to human health, we investigated laying hens, destined to the slaughterhouse, for the presence of acaricide residues in their organs and tissues. We used 45 hens from which we collected a total of 225 samples from the following tissues and organs: skin, fat, liver, muscle, hearth, and kidney. In these samples we analyzed the residual contents of carbaryl and permethrin by LC-MS/MS.

Ninety-one (40.4%) samples were positive to carbaryl and four samples (1.7%) were positive to permethrin. Concentrations of carbaryl exceeding the detection limit (0.005 ppm) were registered in the skin and fat of birds from two farms (p<0.01), although these concentrations remained below the maximum residue limit (MRLs) (0.05 ppm) (p<0.01). All organs/tissues of hens from a third farm were significantly more contaminated, with skin and muscle samples exceeding the MRL (0.05 ppm) (p<0.01) of carbaryl in force before its use was banned. Out of 45 chickens tested, 37 (82.2%) were found to be contaminated by carbaryl, and 4 (8.8%) by permethrin. The present study is the first report on the presence of pesticides banned by the EU (carbaryl) or not licensed for use (permethrin) in the organs and tissues of laying hens, which have been treated against red mites, and then slaughtered for human consumption at the end of their life cycle.

## Introduction

Despite the technological innovations achieved by the poultry industry in recent years and the production rates attained, poultry ectoparasites are of particular concern for the industry [1]. *Dermanyssus gallinae* (De Geer, 1778) (Mesostigmata: Dermanyssidae) is particularly worrying, both for its direct pathogenic effects (obligatory haematophagous mite) and for its role as a vector of bacterial and viral pathogens.

*D. gallinae* has worldwide distribution, and high percentages of infested birds are reported in France, Denmark, Serbia, Montenegro, the Netherlands [2], Sweden [3], Poland [4], UK [5], [6], Romania [7] and in Italy, where the percentage of infested poultry farms reaches 90%.

*D. gallinae* is a less critical problem in the broiler industry due to its short production cycle (52–55 days) [8] but it is a major problem in caged laying hens because of the longer production cycle (10–12 months), and also to the possibility for *D. gallinae* to find more hiding places (egg conveyor belts, transportation cages, walls or floors, hosts' nests, cribs and roosts, dried litter, etc.) and thus to avoid chemical control methods.

Red mites cause itching, and chickens appear nervous and irritable; marked anemia is evident mainly in young subjects, and in extreme cases blood loss due to the mites may lead to death.

Once established on a farm, red mites are almost impossible to eradicate. In the poultry industry, the control of *D. gallinae* red mite primarily relies on acaricide applications, and carbaryl is the most widely used in the past and at present, followed by amitraz, permethrin and organophosphates. The efficacy of these active ingredients against *D. gallinae* is well-documented [9]–[14]. However, despite their proved efficacy against *D. gallinae*, none of these compounds is specifically registered in Italy for use against red mites, except for the very recently labeled organophosphate-based products. This means that farmers have always used - and continue to use - acaricides registered for use in agriculture or for other farm animal species. Due to the absence of compounds specifically labeled for use against red mites, the Veterinary Services has always tolerated the use of these acaricides in the poultry industry, but only when used exclusively between productive cycles and in the absence of birds.

In the last few years, farmers have noticed worldwide that some acaricides have become less effective, and this means that to control mite infestations they are keen to use chemicals at higher concentrations, more frequently and repeatedly - even twice a week, as reported in a recent survey.

This irresponsible behavior may have dangerous consequences for the poultry industry, and also for human health. In fact, the repeated use of acaricides at high concentrations to control infestations could lead firstly to the development of acaricide-resistant *D. gallinae* populations, and more importantly to the accumulation of acaricides in chickens' organs and tissues and also in eggs.

*D. gallinae* strains which are (or are suspected to be) tolerant to acaricides are documented worldwide [10], [12], [15]–[18] including Italy, where a reduced susceptibility to carbamates, pyrethroids, and in part to amidine, has recently been registered in laying farms [19].

EU legislation regulates the detection of pesticides in poultry meat/tissues and eggs; it identifies a limit of residues for each active ingredient, and identifies the MRL for permethrin as 0.05 ppm, which was the same as the level for carbaryl, when its use was still allowed in agriculture and livestock farming. However, due to the methodology used (random sampling; limited classes of acaricides investigated; low numbers of animals controlled) it is possible that some specific/restricted situations of misuse or abuse of chemicals remain undetected.

In order to highlight some situations of risk for human health, we investigated for the presence of acaricide residues in chickens from Italian poultry farms where acaricide-tolerant red mite populations have been found [19], indicating intensive use of chemicals.

## Materials and Methods

### Farms and samples

In 2010, we investigated three farms (denoted A, B and C) in a southern Italian region, and *D. gallinae* populations on all three farms were found to be significantly tolerant to carbammates and permethrins [19]. The farms were medium-sized (about 25,000 animals), and hens were housed in conventional cages. Water came from the public water supply, and commercial feed supplied by a specialized producer was provided *ad libitum*. From spring to the end of October, litter is treated twice a month with cyromazine (Neporex 2WDG) against flies. All three farms perform a continuous production cycle, i.e. without interruption between flock-cycles. Fifteen hens were taken from each farm; they were at the end of their production cycle and destined for slaughter. Since feed may have been contaminated at origin and may have been a possible cause of contamination for chickens, from each farm also feed samples (100 g each for convenience) were collected from their stock of undamaged and previously unopened packs of feed, and one pool of 300 g of feed samples was created.

Animals were transferred to the necropsy laboratory of the Istituto Zooprofilattico of Puglia and Basilicata (Italy).

In the necropsy laboratory, all 45 hens were euthanized using carbon dioxide (CO_2_) and then decapitated. Each bird was placed in an appropriate sealed chamber filled with CO_2_ (70% concentration) and kept in the chamber for several minutes after respiratory arrest. Death was verified by the absence of a detectable heart beat. Decapitation was performed using appropriate equipment. Since animals react adversely to the smell of blood, decapitation was not performed in the presence of other animals, and the operator changed gloves and washed hands between decapitations. Samples from liver, fat, skin, muscle, and kidney plus heart were collected from each animal resulting in a total of 225 samples. For the control animals, the same organs and tissues were collected from a newborn chick whose death was due to non-pathological causes. All tissues and organs collected were immediately and individually placed in single transparent bags, properly labeled and kept at −80°C until successive processing.

All the experimental procedures met the Italian National Laws (*Decreto Legislativo* 116/92), the European Communities Council Directive (86/609/EEC) and were performed following the Guidelines for Animal Care and Use of the National Institutes of Health. The study was approved by the Italian Ministry of Health (permit number 46, prot. 475 at the Istituto Zooprofilattico of Puglia and Basilicata). All efforts were made to minimize the number of animals used in the study and their suffering.

### Chemical and Reagents

Solvents (methanol, acetonitrile), formic acid, ammonium formiate, and standard acaricides (carbaryl and permethrin) were acquired from Sigma-Aldrich (St. Louis, MO, USA). Agilent Technologies (Palo Alto, CA, USA) provided the PTFE membranes (0,45 µm) used to filter the extracts before injection into the chromatographic system. Unless otherwise indicated, all reagents used in the study were HPLC-grade and analytically pure substances. Pure water was generated by a Milli-Q water–purification system (Millipore, Bedford, MA, USA).

### Standard solutions

The individual stock solution of carbaryl and permethrin was prepared by dissolving 450 mg of carbaryl and 731.6 mg of permethrin in 1 mL of acetonitrile; this was then stored at −20°C. Similarly, mixed working standard solutions were prepared by diluting the stock solutions in methanol and these were then stored at 4°C.

### Sample extraction and cleanup using QuEChERS methods

The heart and kidneys from each bird were processed together to achieve the minimum weight needed for analysis. Approximately 10 g of each animal organ/tissue sample was minced using a kitchen liquidizer, and then stored at −20°C before use in the experiments. Equipment was carefully rinsed with water and acetonitrile between processing of samples. QuEChERS (Quick, Easy, Cheap, Effective, Rugged, and Safe) extraction was performed using disposable 50 mL extraction tubes containing 4 g of MgSO_4_, 1 g of sodium citrate, 0.5 g of sodium hydrogencitrate sesquihydrate and 1 g of sodium chloride (Agilent Technologies, Palo Alto, CA, USA). The sample was mixed with 10 ml of acetonitrile and centrifuged for 5 minutes at 2.500 g. The supernatant was cleaned by dispersive solid-phase extraction (dSPE, Silica, 100 mg SampliQ Solid Phase Extraction) (Agilent Technologies) and centrifuged as before. Finally, the extract was filtered and injected into LC-MS/MS for analysis.

A sub-pooled sample of 10 g of feed was created and directly subjected to extraction as described above. The extraction procedure was carried out in duplicate for each sample.

### LC-MS/MS analysis

Analysis was carried out using a High Performance Liquid Chromatograph (Agilent Technologies 1200 Series) coupled to an Agilent QQQ Triple Quadrupole Mass Detector (mod. 6410°2 K) and an Agilent Mod. G1367C autosampler. Separation was achieved using a Zorbax Eclipse Plus RRHT C18 column (100 mm length×2.1 mm inner diameter) filled with 1.8 µm diameter particles as the stationary phase (column operating temperature set at 40°C). The mobile phase was composed of an aqueous solution of 5 mM ammonium formiate/0.1% formic acid (A) and acetonitrile/methanol 50/50 v/v (B). The gradient was run as follows: 0.3 min A 100%; from 0% to 35% B in 3 min; from 35% to 65% B in 22 min; and from 65% to 100% B in 10 min. The flow rate was 0.3 mL/min and injection volume was 5 µl. The QQQ mass detector was equipped with an electrospray interface, operating in positive ion mode with the following parameters: source voltage 4 kV, capillary temperature 350°C, sheath gas (N_2_) 40 psi, auxiliary gas (N_2_) 5 psi, and collision gas (N_2_) 1.5 m Torr. Multiple reaction monitoring (MRM) was performed on each analyte by choosing two product ions from a precursor ion. The collision energy values ranged from 15 to 30 eV and were optimized to maximize product ion intensity, obtaining precursor ion intensities around 10% (normalized intensity).

In LC-MS/MS analysis, peaks were identified by comparing retention times, precursor and product ions with those relevant to standards analyzed under the same operating conditions. LC-MS/MS information for the target analytes is as follows: retention time for carbaryl was 11 min, the precursor ion was at 202.0 m/z, and product ions were at 145.0 and 127.0 m/z. Retention time for permethrin was 29 min, the precursor ion was at 408.0 m/z, and product ions were at 355.0 and 183.0 m/z.

### Method validation

A calibration curve was obtained by injecting solutions with variable amounts of standards in order to cover the desired concentration range.

Recovery analyses were carried out on all the uncontaminated matrices spiked at 0.1 mg/kg of pesticide standards. After sample preparation, aliquots were analyzed according to the proposed method. The recovery values were calculated as the ratio between the observed and spiked concentrations. Finally, the residue concentrations were obtained using the calibration curve and dividing the calculated concentrations by the corresponding recovery factor. The final data were reported in mg/kg (ppm) on fat basis. Repeatability was calculated as the relative standard deviation obtained by determining analytes concentration in eight uncontaminated skin samples spiked at 0.005 ppm.

The limits of detection (LODs) were calculated as the concentration corresponding to a signal to noise (S/N) ratio of 3. All analyses were carried out in duplicate; control analyses were also performed in order to check interference from the sample. LODs, and average recoveries for carbaryl and permethrin are shown in **Table 1**.

**Table 1:** Detection limits (LOD) and the average recoveries (± SD) of carbaryl and permethrin for all matrices.

PESTICIDES(LOD PPM)	PERCENTAGE OF RECOVERY					
	Fat	Muscle	Liver	Skin	HK	Feed
**Carbaryl (0.005)**	85.3±3.7	88.7±11.3	92.6±2.1	81.1±1.9	90.5±1.6	78.0+−1.2
**Permethrin (0.005)**	80.3±0.6	81.1±1.9	83.5±0.6	76.2±1.1	83.7±2.9	77.0+−1.1

**HK**: Heart and Kidney.

### Statistical analysis

Data obtained from tissues/organs of animals from the same farm were considered as belonging to the same statistical population, since all animals from each farm were bred and sampled in the same way. Data collected from the duplicate extractions were averaged, therefore a sample set (n = 15) were obtained and processed by one-way variance analysis (ANOVA), with 99% confidence levels. Duncan's test was used to determine statistically significant differences between tissues/organs within each farm and between farms. Finally, one-tailed t-student test, with a 99% confidence level, was used to verify the statistical hypothesis X_mean_>μ_0_, where X_mean_ is the mean of concentration values and μ_0_ is the maximum residue limit (MRLs) in force when carbaryl use was still legal in agriculture and livestock farming (0.05 ppm). The t-critical value was 2.62 at 14 degrees of freedom and α = 0.01. The Statistica 6.0 software package was used.

## Results

Out of 45 laying hens from three different poultry farms, 37 (82.2%) were positive for carbaryl residues and 4 (8.8%) for permethrin (**Table 2** **)**. Out of 225 samples obtained, 91 (40.4%) samples resulted positive for carbaryl (25 skin, 27 fat, 8 liver, 16 muscle, 15 heart and kidney samples), showing a mean concentration of 5 ppm, 0.04 ppm, 0.05 ppm, 0.14 ppm, 0.04 ppm, respectively (**Table 2**). Four samples (1.7%) resulted positive for permethrin (2 fat and 2 liver samples) (**Table 2**), with a mean concentration of 0.012 ppm and 0.006 ppm, respectively (**Table 2**). On one farm (Farm B), all investigated hens were found to be contaminated by carbaryl (**Table 2**), and 80% of their organs and tissues contained residues of the compound (**Table 2**), with the highest concentrations in the skin (16 ppm), fat (0.11 ppm) and muscle (0.3 ppm) (**Table 2**).

**Table 2:** Number, percentage (%) and mean concentrations (ppm) of positive organs/tissues and number of chickens positive to carbaryl and permethrin from Farms A, B and C.

	FARM A		FARM B		FARM C		TOTAL	
	C(%)/Mc	P(%)/Mc	C(%)/Mc	P(%)/Mc	C(%)/Mc	P(%)/Mc	C(%)/Mc	P(%)/Mc
**Skin**	9/15(60)/0.013	0/15(0)	10/15(66.6)/16	0/15(0)	6/15(40)/0.01	0/15(0)	25/45(55.5)/5	0/45
**Fat**	8/15(53.3/0.009	2/15(13.3)/0.012	13/15(86.6)/0.11	0/15	6/15(40)/0.009	0/15	27/45 (60)/0.04	2/45(4.4)/0.012
**Liver**	1/15(6.6)/0.05	2/15(13.3)/0.006	7/15 (46.6)/0.04	0/15	0/15	0/15	8/45 (17.7)/0.05	2/45(4.4)/0.006
**Muscle**	0/15(0)	0/15 (0)	15/15(100)/0.3	0/15	1/15(6.6)/0.006	0/15	16/45(35.5)/0.14	0/45
**HK**	0/15(0)	0/15(0)	15/15(100)/0.04	0/15	0/15	0/15	15/45(33.3)/0.04	0/45
**TOTAL**	18/75(24)	4/75(5.3)	60/75(80)	0/75	13/75(17.3)	0/75	91/225 (40.4)	4/225 (1.7)
**No P/T A** *	13/15(86.6)	4/15(26.6)	15/15(100)		9/15(60)	0/15	37/45(82.2)	4/45(8.8)

**C** = Carbaryl; **P** = Permethrin; **Mc:** Mean concentration of positives (ppm); **HK**: Heart and Kidney.

**No P/T A:** Number of Positive/Tested Animals in percentage.

* Animals were considered positive when at least one organ/tissue was found positive to the investigated acaricides.

Statistical analysis was performed only on data obtained for carbaryl, because the number of positive samples for permethrin was too low to allow data treatment.

**Table 3** shows the comparison of tissues/organs within each farm and between farms, for each tissue/organ (ANOVA), while **Table 4** shows the comparison between the results obtained and the maximum residue limit (MRLs) in force when carbaryl use was still legal for agriculture and livestock (0.05 ppm) (National Residues Plan 2007). Carbaryl concentrations higher than or equal to the detection limit were registered in the skin and fat of hens from Farms A and C (p<0.01); however, these were below the maximum residue limits (MRLs) (p<0.01). All organs/tissues from Farm B were found to be significantly more contaminated than those from the other farms (p<0.01), with skin showing the highest concentrations. In addition, skin and muscle samples from Farm B exceeded the maximum residue limits (MRLs) (p<0.01). **Table 4** shows all the statistical parameters (level range, median, mean, quartiles, standard deviation, standard error and t-value) from all the investigated farms. Data showed a large variability among the investigated farms and organs/tissues, whereas repeatability of analytical method was 0.00007 ppm. Farm B median values indicate that 50% of organs/tissues presented carbaryl concentrations, which were higher than, or equal to, 0.005 (detection limit). Specifically, carbaryl concentrations exceeded 14 ppm in skin samples; 0.17 ppm in muscle samples; 0.04 ppm in fat samples; 0.02 ppm in heart and kidney samples; and 0.005 ppm in liver samples (**Table 4**).

**Table 3:** ANOVA results for data obtained from carbaryl HPLC-MS analysis in chicken organs/tissues from Farms A, B and C.

	FARM A		FARM B		FARM C	
	Concentration Mean		Concentration Mean		Concentration Mean	
	C	P	C	P	C	P
**Skin**	0.009^a^ ^A^	ND	11^a^ ^B^	ND	0.007^a^ ^A^	ND
**Fat**	0.006^a^ ^A^	ND	0.10^b^ ^B^	ND	0.005^a^ ^A^	ND
**Liver**	ND	ND	0.02^b^	ND	ND	ND
**Muscle**	ND	ND	0.3^b^	ND	ND	ND
**H&K**	ND	ND	0.04^b^	ND	ND	ND

**C** = Carbaryl; **P** = Permethrin; **H&K**: Heart and Kidney.

a,b Means in the same column followed by different small letters differ significantly (One-way variance analysis, P<0.01).

A,B Means in the same row followed by different capital letters differ significantly (One-way variance analysis, P<0.01).

**ND**: Concentrations found below the detection limit (0.005 ppm).

**Table 4:** Statistical parameters of data obtained from HPLC-MS analysis of carbaryl in 45 chicken organs/tissues from Farms A, B and C.

	FARM A					FARM B					FARM C				
	Skin	Fat	Liver	Muscle	HK	Skin	Fat	Liver	Muscle	HK	Skin	Fat	Liver	Muscle	HK
LR*	ND–0.037	ND-0.015	ND-0.005	ND	ND	ND-26	ND-0.42	ND-0.25	0.020–0.69	0.005–0.15	ND-0.023	ND-0.012	ND	ND-0.006	ND
Median*	0.007	0.005	ND	ND	ND	14	0.04	0.005	0.17	0.02	0.004	0.0041	ND	ND	ND
Q1*	ND	ND	ND	ND	ND	0	0.03	ND	0.12	0.016	ND	ND	ND	ND	ND
Q3*	0.012	0.008	ND	ND	ND	17	0.15	0.009	0.37	0.03	0.012	0.008	ND	ND	ND
Mean*	0.009	0.006	ND	ND	ND	11	0.10	0.02	0.3	0.04	0.007	0.005	ND	ND	ND
SD	0.009	0.005	-	-	-	9	0.13	0.06	0.2	0.04	0.007	0.004	-	-	-
SE	0.002	0.0013	-	-	-	2	0.03	0.017	0.05	0.011	0.0017	0.0011	-	-	-
t-value**	-	-	-	-	-	4.55	1.43	-	3.92	-	-	-	-	-	-

**LR:** Level Range; **HK**: Heart and Kidney; **ND**: Not Detected (concentration values below detection limit (0.005 ppm).

**SD:** Standard deviation; **SE**: Standard error;

* All the values are in ppm.

** t-value has been calculated for mean concentrations higher than or equal to MRL (0.05 ppm).

All organs and tissues from newborn chicks (control) and feed samples tested negative for both carbaryl and permethrin (detection limit: 0.005 ppm).

## Discussion

This study shows that most laying hens (37 out of 45) from all three investigated farms were contaminated by carbaryl, and that the hens of one farm also contained permethrin. Furthermore, with different accumulation levels among animals – possibly due to differences in factors like management strategies and unpredictable individual predispositions - all organs/tissues were contaminated by carbaryl, with the highest levels found in skin, fat, and muscle (**Table 2**).

These data are all worrying, because: *a)* carbaryl was banned by the EU in 2007 (Allegato I, Direttiva 91/414, 1376/07, 07/355); *b)* no carbaryl-based products specifically labeled for use against *D. gallinae* infestation were available on the Italian market before the ban; *c)* no registered permethrin-based products are available on the market for use against red mite infestation; and *d)* tissues and organs from laying hens can be consumed as food.

Several compounds have proved effective against *D. gallinae in vitro* and *in vivo* trials i.e. carbaryl [10], bendiocard [10], dichlorvos [10], [12], triclorphon [13], tetraclorvinphos, pirimiphos methyl [11], phoxim [14], flumethrin [9], permethrin [10], [17], fenvalerate [10], cyalotrin ([11], and amitraz [10]. However, it is only very recently (late 2010) that active ingredients specifically registered for use against *D. gallinae* have become available on the Italian market: a phoxim-based (ByeMite® BAYER), and a spinosad-based product (Elector® ELANCO).

The data obtained in this study reflect the history and consequences of extensive and improper use of unlicensed pesticides (high concentrations and frequency of application). In fact, heavy chemical pressure may cause mortality of sensitive individual red mites and the survival of some resistant individuals; in this way, a new generation of resistant individuals develops. On the other hand, chemicals may accumulate in chicken skin, fat, liver, kidneys, and also in eggs.

Red mite populations resistant to several compounds have been reported worldwide. In the former Czech Republic, strains of *D. gallinae* were found to be resistant to DDT, but also possibly to permethrin, tetramethrin and trichlorphon [10]. In France, Beugnet [10] reported reduced effectiveness of permethrin and diclorvos against red mite, and the authors attributed this to repeated use of these compounds by farmers. Other contributions on the ineffectiveness of acaricides in field conditions are also recorded in Germany [16], Sweden [17], UK [5], and Hungary [18]. When seven Italian farms were investigated recently, red mite field populations were found to be tolerant - even at their highest concentrations - to carbaryl on six farms (86%) and to permethrin on three farms (42%) (P<0.05) [19].

Over 90% of human exposure to pesticides is caused by the consumption of contaminated food, mainly of animal origin (meat or fish) [20]. Farmed animals can take in pesticides through contaminated feeds of animal or plant origin, or through veterinary products used to control parasite infestations [21]–[24].

In the present study, the presence of acaricides in organ and tissues of laying hens seems unequivocally due to the chemical pressure applied by farmers, for the following reasons: *a)* red mite populations unsusceptible/resistant to carbaryl and permethrin were registered on the same farms [19]; *b)* farmers have confirmed their repeated use of these compounds against red mites; *c)* feed provided to animals and tested in the present study resulted negative to acaricides.

It is known that in countries where large-scale use or abuse of pesticides is a common practice, there is a high risk of consumers accumulating chemicals [25], [26]. Surveys on the presence of chemicals in different animal species were recently reviewed [27]. In Jordan, out of 115 chicken samples tested, 20% contained organochlorine compounds [28], and the same compounds have been reported in poultry meat in China [29]. Problems related to residues also involve European countries; meat samples from chickens experimentally treated with organophosphate (propetamphos) and pyrethroid (permethrin) compounds available on the market in Hungary [30] tested positive only to organophosphates; no residues of permethrin were found with a detection limit of 0.01 ppm. A report from the UK states that residues of carbaryl and its metabolites have been detected in eggs; according to the authors this contamination was related to pesticides used against mites [31]. Thus, the present study is the first report on the presence of permethrin and carbaryl in poultry organs and tissues (detection limit of 0.005 ppm).

Due to the absence of compounds specifically labeled for use against red mites, the use of permethrin and carbaryl has always been tolerated by the Italian Veterinary Service; however, despite the rules that they should be used only between flock-cycles in the absence of animals, our findings confirm that farmers have always used - and continue to use – acaricides registered for use in agriculture or for other livestock species. More importantly, our findings confirm that these are commonly applied when the birds are present. In addition, carbaryl was banned in 2007, and is therefore being used illegally.

The significant highest concentration of residues found on one farm (much higher than MLRs in force when carbaryl use was legal) document very recent treatment carried out by the farmers, and may be related to the lack of a break between two flock-cycles, i.e. the coexistence of young hens (15–16 weeks) and old hens (40–60 weeks) at the end of their flock-cycle.

The results obtained from all farms (**Tables 3** **and** **4**) show, as expected, that skin and fat are the tissues at greatest risk of accumulation because of their highly lipophilic structure and because of acaricide stability; therefore they pose the greatest risk for human health. However, muscle can also be at even more risk than fat, as shown in the very recently treated animals i.e. those bred on Farm B (**Tables 3** **and** **4**).

These data are alarming if we consider the toxic effects of pesticide accumulation on human health. Pregnant women run the greatest risk; several contributions have documented the passage of acaricides to newborns in maternal milk, or through the umbilical cord to the fetus [32]–[33], their accumulation in the placenta and fetal liver [34] with the consequent risk of premature deliveries, and the birth of underweight and/or congenitally malformed babies [35]. Exposure to acaricides seems also to be associated with several other health risks i.e. cardio- circulatory diseases and infarction [36], prostate cancer [37], carcinoma testis of germinal cells [38], genetic mutations [39], brain damage, neurotoxic disorders [40], and a state of severe depression in young people when continuously exposed to pesticides [41].

In conclusion, the present study is the first report in Europe on the presence of pesticides in the organs and tissues of poultry treated against red mites, which are often commercialized at the end of their production cycle (about 12 months) for use in ‘chicken broth’.

The detection of acaricide residues in tissues/organs of laying hens seems to confirm - at least in the studied area - their extensive and improper use by farmers against *D. gallinae*. It also shows up the illegal use and persistent commercialization of pesticides banned years ago (carbaryl), and more importantly, it indicates that some specific/restricted situations of misuse or abuse of chemicals may remain undetectable.

Misuse/abuse of chemicals may actually be more widespread in Italy, and a larger number of farms should be investigated in order to acquire a realistic estimate of the extent of illegal practice. However, the data presented here have at least made it possible to highlight some situations in areas where sanitary management is poor and unsupervised by specialized technicians. The current availability on the Italian market of products specifically licensed for use against *D. gallinae* may help farmers to manage infestations better and to limit the consequences related to misuse of chemicals.

In order to ensure a correct integrated control strategy, until better alternative control methods are developed, farmers should use acaricides appropriately. This means using only licensed products after first testing their efficacy; rotating the compounds used; and applying only the correct concentrations and formulations. In the mean time, National Health Authorities should ensure that farmers use the appropriate chemicals correctly. These measures are vital for farmers and consumers alike, to reduce the risk that resistant red mite populations will proliferate, and to ensure that meat and egg products are safe to eat.
